# Short-Term Traffic State Prediction Based on the Critical Road Selection Optimization in Transportation Networks

**DOI:** 10.1155/2021/9966382

**Published:** 2021-08-30

**Authors:** Tian Ma, Guanghong Gong, Yilong Ren

**Affiliations:** ^1^School of Automation Science and Electrical Engineering, Beihang University, Beijing 100191, China; ^2^School of Transportation Science and Engineering, Beihang University, Beijing 100191, China

## Abstract

Short-term traffic prediction under corrupted or missing data for large-scale transportation networks has become an important and challenging topic in recent decades. Since the critical roads have predictive power on their adjacent roads, this paper proposes a novel hybrid short-term traffic state prediction method based on critical road selection optimization. First, the utility function of the quality of service (QoS) for the critical roads in a large-scale road network is proposed based on the coverage and the data score. Then, the critical road selection optimization model in the transportation networks is presented by selecting an appropriate set of critical roads with the maximum proportion of the total calculation resources to maximize the utility value of the QoS. Also, an innovative critical road selection method is introduced, which is considering the topological structure and the mobility of the urban road network. Subsequently, the traffic speed of the critical roads is regarded as the input of the convolutional long short-term memory neural network to predict the future traffic states of the entire network. Experiment results on the Beijing traffic network indicate that the proposed method outperforms prevailing DL approaches in the case of considering critical road sections.

## 1. Introduction

Real-time traffic state prediction plays a vital role in traffic management and public service. By predicting the evolution of traffic timely and accurately, governments and travelers could react to the traffic congestion ahead of time. For instance, intelligent transportation systems, advanced traffic management systems, and traveler information systems depend on real-time traffic state prediction.

In the past decades, there have been numerous studies on this topic [1]. These studies could be divided into mathematical models, statistical models, and data-driven methods [2]. Compared with data-driven methods, mathematical or statistical models derived from macroscopic and microscopic theories of traffic flow are difficult to handle unstable traffic conditions and complex road settings due to strong hypotheses and assumptions [3].

Data-driven methods have achieved promising results due to more potential in processing complex nonlinear problems [4]. These methods include support vector machine (SVM), Bayesian network, and neural network. Among all these data-driven methods, deep learning approaches have proven effective in traffic state prediction. This method could exploit much deeper architectures and process the high-dimensional set of explanatory variables [5].

However, most of the deep learning approaches are constructed based on the entire dataset. The attributes of datasets influence the prediction performance. In other words, the deep learning approaches have highlighted the data quality in short-term traffic state prediction [5]. Due to the corrupted or missing data problem, there is limited high-quality real-time or historical data obtained, indicating that the data has low predictive quality [6]. These setbacks weaken the predictive accuracy and efficiency, limiting the capacity for providing a practical and reliable forecasting result.

Recently, researchers find that some critical roads significantly affect the traffic states of their adjacent roads at a specific road network [7, 8]. This conclusion indicates that the traffic state of one road could be predicted based on its neighbors' state [6].

There have been numerous studies on this topic, but only a tiny percentage of them have paid attention to prediction based on critical road selection optimization. Therefore, if we extract the traffic state of the critical road sections with the most dominant predictive power, we could characterize the spatiotemporal features of traffic flow and predict the future traffic state of the overall network.

In this paper, we propose a novel hybrid short-term traffic state prediction method based on critical road selection optimization. Different scores were given to data collected on different road segments. The higher the criticality of the road segment, the higher the score of the data. The critical road selection problem is abstracted as a multiobjective optimization problem, maximizing the sensing coverage and data scores. In other words, our objective is to select the most suitable critical roads to maximize the quality of the service (QoS) with the limited consumption of network resources.

Then, a novel critical road selection method is proposed, considering the topological structure and the mobility of the urban road network. Subsequently, the traffic speed of the critical roads is regarded as the input of the convolutional long short-term memory neural network to predict the future traffic states of the entire network. Finally, to demonstrate the effectiveness of the proposed method, the numerical experiments using the traffic states depicted from GPS trajectory data in Beijing. In addition, other traditional machine-learning models are compared to demonstrate the advantage of the proposed method. Practical experiment results showed that the proposed method could precisely predict future traffic network states.

The rest of our paper is organized as follows.  Section 2 discusses the literature on short-term traffic state prediction and the existing approaches to prediction based on critical roads. In Section 3, the critical road selection optimization model is proposed by selecting an appropriate set of critical roads with the maximum proportion of the total calculation resources to maximize the utility value of the QoS and also an innovative critical road selection method is introduced.  Section 4 elaborates on the numerical experiments using the traffic states depicted from GPS trajectory data in Beijing. The last section concludes the study and discusses future work.

## 2. Literature Review

Over the past decades, considerable short-term traffic forecast models have emerged to handle the prediction of future traffic states ranging from a few seconds to few hours. These approaches could be generally categorized into mathematical approaches, statistical approaches, and data-driven approaches.

Mathematical approaches focus on predetermining the model structure by theoretical assumption. The evolution of the traffic state could be simulated by the theoretical mathematical models [9]. Because of the strong dependence on theoretical considerations, these mathematical approaches do not match the actual traffic state condition [10]. Mathematical approaches depend on theoretical mathematical models to simulate the traffic evolution. There are many famous mathematical models in the past decades, such as the Greenshields model, car-following model, Van Lighthill–Whitham–Richards (LWR) model, and so on. The future traffic state of the road network could be calculated by these models directly [11, 12]. Most traffic simulation simulators, such as Q-Paramics, VISSIM, DynaMIT, and DynaSMART-X, predict traffic states based on the traffic flow models, car-following models, and dynamic traffic assignment models [13–16].

Statistical approaches usually rely on statistical assumptions. The autoregressive integrated moving average (ARIMA) and its variants are the most common mathematical approaches. Hamed et al. [17] proposed a simple ARIMA to predict the traffic state of the road network. Williams et al. developed a seasonal ARIMA (S-ARIMA) to predict the traffic state of the urban freeway. The results showed that the S-ARIMA model could obtain better properties [18, 19]. Ding et al. proposed a space-time ARIMA to predict the traffic state of the road network [20].

In addition, the Markov chain, Kalman filter (KF), KF-based approaches, and other approaches also have important applications in short-term traffic prediction [21–24]. However, these approaches fail to produce favorable results under unstable traffic conditions, such as unexpected events [25].

Different from mathematical approaches and statistical approaches, data-driven approaches rely on a sufficient mass of traffic data. In recent years, due to abundant data attached to extensive traffic sensors and advanced big data technology, data-driven approaches have developed rapidly. Numerous data-driven approaches were put forward for the short time traffic state prediction, such as SVM [26–28], neural network [29–32], and hybrid methods [33, 34].

Among these data-driven approaches, deep learning methods have become extremely popular and successful because of their powerful ability to process nonlinear high-dimensional problems. Huang et al. employed a deep belief network (DBN) with multitask learning for traffic flow prediction [4]. Lv et al. proposed an SAE model to predict the traffic flow, and the performance is superior to other methods at different prediction horizons [35]. Furthermore, numerous efforts have been devoted to emphasizing the temporal characteristics and spatial dependencies on prediction [2]. Ma et al. predicted the traffic speed of a large-scale transportation network using an LSTM neural network and CNN [36, 37]. Wu and Tan extracted spatial and temporal features by CNN and LSTM, respectively, and predicted traffic volume combined these two approaches [38]. Wang et al. proposed an eRCNN model then trained the recurrent CNN by reducing predictive feedback errors [39].

In summary, among all these traffic state prediction approaches, deep learning methods stand out as the most potent alternative. However, few prediction methods could achieve satisfactory accuracy because of the missing data problem in reality. For the critical roads that have a significant effect on the traffic states of their respectively adjacent roads at a specific road network, we could extract the traffic state of the critical road sections and predict the future traffic state of the overall network.

## 3. Methodology

This research focuses on utilizing data from critical road sections to predict future traffic conditions of the overall urban transportation network. In this section, the utility function of the QoS for the critical roads in a large-scale road network is proposed based on the coverage and the data score. Then, the critical road selection optimization in the transportation networks is presented by selecting an appropriate set of critical roads with the maximum proportion of the total calculation resources to maximize the utility value of the QoS. Specifically, the critical road sections are selected by an innovative critical road selection method. Finally, the traffic speed of the critical roads is regarded as the input of the convolutional long short-term memory neural network to predict the future traffic states of the entire network.

### 3.1. Road Network Topology Analysis

In the practical urban road network, road sections are connected at intersections and eventually form a complex network. When performing sensing tasks in urban road network areas, the topological structure characteristics of the road network need to be considered. The results of numerous studies have shown that the topology of urban road networks is complex and diverse. The failure of connectivity in some sections of the network can impact the traffic operation in the whole network. However, it is inevitable that road connectivity in the network will sometimes be interrupted due to bad weather, technical failures, or serious accidents. This will lead to local traffic congestion and paralysis in the network, which will have harmful economic and social impacts. It means that the higher importance of road sections in the network under different spatial and temporal conditions indicates the more severe damage to the integrity of the road network connectivity brought by their failure. In order to avoid serious impacts on road network connectivity and vehicle movements, priority should be given to the use of high, critically important road sections for future traffic state prediction.

In order to study the structural properties of real road networks, it is necessary to reasonably abstract the road networks into topological structure diagrams, consisting of points and lines by suitable methods. The primal approach and the dual approach are two methods to abstract the road network into a complex network model. The primal approach uses the roads in the road network as edges in the abstract network and the intersections as nodes in the abstract network. The dual approach models the intersections as edges in the network and the roads in the urban road network as nodes, thus showing the interconnections between roads in a highly abstract way. The primal approach is intuitive and simple and can retain the layout characteristics of the road network. The dual approach ignores some geographic significance of network entities, such as the geographic location of roads, length, and width, and therefore, it is more suitable for analyzing abstract network structures. In this paper, we pay more attention to the characteristics of road connectivity, so we use the primal approach to model the road network.

### 3.2. QoS for the Critical Roads

The QoS is the standard for measuring the performance of the critical roads in a prediction task. The greater the value of QoS, the better the prediction performance of the critical roads. Here, we propose a utility function to calculate the QoS for the critical roads.

The coverage of the selected roads is mainly concerned with people when predicting the traffic state of the whole road network. So, we choose coverage as our first metric. Coverage indicates the coverage of the selected vehicle to the entire road network. For better calculating the coverage *C*, we divide the road network into small grids, and the grid is used as the basic measuring element for coverage calculation. As shown in Figure 1, the pink curves represent roads. The grid with roads passing through is painted green. In this paper, the size of the grid is 0.0005° × 0.0005°, based on longitude and latitude, where 0.0005 longitude (latitude) is about 50 m.

Define *g*_*j*_ as the single grid in the urban road network. Let *f*(*g*_*j*_) represent the coverage state of *g*_*j*_, and *f*(*g*_*j*_)=1 indicates that grid *j* is selected during the predicting task time; otherwise, *f*(*g*_*j*_)=0. In this paper, we tried to predict the whole network traffic state. If *g*_*j*_ belongs to road section *l* and road section *l* has *φ* grids, then the road factors could be calculated as ∂(*g*_*j*_)=1/*φ*. The following equations could calculate the coverage of the selected grids:

(1) $$\begin{array}{c} f\left(g_{j}\right)=\left\{\begin{array}{cc} 1, & \text{if }g_{j}\text{ is selected in predicting task,}\\ 0, & \text{otherwise}, \end{array}\right.\\ C=\frac{\sum_{i=1}^{n}f\left(g_{j}\right)*\partial \left(g_{j}\right)}{n}. \end{array}$$

On the other hand, we introduce the concept of data score to represent the criticality level of the roads. Specially, we give a higher score to the data collected from the critical roads than the data collected from the ordinary roads. Here, we use the correlations among road sections on both space and time to calculate the data score.

The spatial weights matrix represents the spatial dependency among road sections in traffic networks. According to graph theory, the local connectivity of a node can be calculated based on the connection between the node and its adjacent node, which is represented by the degree of node *k*. Suppose there exists a network, which can be represented as *G*=(*V*′, *E*), where *V*′ is the set of nodes in the network and *E* is the set of edges in the network, representing the connections between nodes in the network. The network *G*=(*V*′, *E*) has |*V*′|=*N* nodes and |*E*|=*M* edges. Then, this network can be represented by the adjacency matrix *A*_*M*×*N*_. If nodes *i* and *j* are connected directly or indirectly, we call these two nodes “*k*th-order neighbors,” and their adjacency relationship could be expressed as equation (2). The spatial weights matrix *P* could be defined as the sum of the *k*th spatial weights matrix; element *p*_*ij*_ in *P* is calculated as shown in equation (3).

(2) $$\begin{array}{c} A_{ij}^{k}=\left\{\begin{array}{cc} 1, & \text{when nodes }i\text{ and }j\text{ are directly connected},\\ 0, & \text{otherwise,} \end{array}\right. \end{array}$$

(3) $$\begin{array}{c} p_{ij}=\sum_{i=1}^{K}\sum_{j\neq i}^{n}A_{ij}^{k}, \end{array}$$

where *K* is the highest order of the spatial weights matrix.

And, to comprehensively consider the spatial correlation of the road network with the temporal correlation, the spatial weights matrix is introduced as a spatial indicator to improve the initial correlation distance. Let *x*_*i*_^*t*^ be traffic speed in the road section *i* at time *t*, where *x*_*i*_^*t*^=(*x*_*i*_^1^, *x*_*i*_^2^,…, *x*_*i*_^*T*^). Then, the integrated speed values of the adjacent road sections RX_*i*_^*t*^ could be computed by equation (4). Then, the data score *D*_*i*_(*s*) between road section *i* and its adjacent road sections could be calculated by equation (5):

(4) $$\begin{array}{c} {\text{RX}}_{i}^{t}=\sum_{j=1}^{R}P_{ij}x_{j}^{t}, \end{array}$$

(5) $$\begin{array}{c} D_{i}\left(s\right)=1-\frac{\sum_{t=1}^{T}\left(x_{i}^{t}-\bar{x_{i}}\right)\left({\text{RX}}_{i}^{t+s}-\bar{{\text{RX}}_{i}}\right)}{\sqrt{\sum_{t=1}^{T}{\left(x_{i}^{t}-\bar{x_{i}}\right)}^{2}}\sqrt{\sum_{t=1}^{T}\left({\text{RX}}_{i}^{t+s}-\bar{{\text{RX}}_{i}}\right)}}, \end{array}$$

where *s*=(1,2,…, *S*) (*s* > 0) is the time lag between the speeds of road sections *i* and its adjacent road sections; $\bar{x_{i}}$ is the mean value of traffic speed *x*_*i*_^*t*^ in road sections *i* during the time duration of *T*. $\bar{{\text{RX}}_{i}}$ is the mean value of integrated speed RX_*i*_^*t*^. Based on the previous analysis, mathematical expressions of data score *D* are defined as follows:

(6) $$\begin{array}{c} D=\sum_{i=1}^{n}D_{i}\left(s\right)\text{.} \end{array}$$

The utility function of QoS, *U*, is defined as

(7) $$\begin{array}{c} U=\alpha \cdot \;\log_{2}\;C+\left(1-\alpha \right)\cdot \;\ln\;D, \end{array}$$

where *α* ∈ [0,1] is a parameter for tuning the weight of data coverage and data score. To make *α* more sensitive in equation (7), we apply log_2_*C* instead of *C* and ln  *D* instead of *D*. Since logarithm is a common way to aggregate data, this process can reduce the heteroscedasticity of data in the QoS function.

### 3.3. The Critical Road Selection Optimization

#### 3.3.1. Definition of the Critical Road Selection Problem

The goal of the critical road selection model is to maximize the QoS of the urban traffic prediction system with limited critical roads, so the mathematical expression of the critical roads selection problem can be defined as

(8) $$\begin{array}{c} \max U=\alpha \cdot \;\log_{2}\;C+\left(1-\alpha \right)\cdot \;\ln\sum_{j=1}^{n}D_{i}\left(s\right)\\ \text{s.t.}\;\left\{\begin{array}{c} C=\frac{\sum_{i=1}^{n}f\left(g_{j}\right)*\;\partial \left(g_{j}\right)}{n},\\ f\left(g_{j}\right)=\left\{\begin{array}{cc} 1, & \text{if }g_{j}\text{ is selected in predicting task},\\ 0, & \text{otherwise,} \end{array}\right.\\ F=\left\{f\left(g_{j}\right)|i=1,2,\ldots ,n\right\},\\ 0\leq \alpha \leq 1,\\ D_{i}\left(s\right)=1-\frac{\sum_{t=1}^{T}\left(x_{i}^{t}-\bar{x_{i}}\right)\left({\text{RX}}_{i}^{t+s}-\bar{{\text{RX}}_{i}}\right)}{\sqrt{\sum_{t=1}^{T}{\left(x_{i}^{t}-\bar{x_{i}}\right)}^{2}}\sqrt{\sum_{t=1}^{T}\left({\text{RX}}_{i}^{t+s}-\bar{{\text{RX}}_{i}}\right)}},\\ x_{i}^{t}=\left(x_{i}^{1},x_{i}^{2},\ldots ,x_{i}^{T}\right),\\ \partial \left(g_{j}\right)=\frac{1}{\varphi },\\ C<\mu , \end{array}\right. \end{array}$$

where function *U* is used to calculate the utility value of the QoS; *f*(*g*_*j*_) represents whether grid *j* is selected, with *f*(*g*_*j*_)=1 indicating that grid *j* has been selected; otherwise, the value of *f*(*g*_*j*_) is 0. *F* is the set of critical roads, and *C* is the coverage. *D*_*i*_(*s*) is the data score between road section *i* and its adjacent road sections. *μ* is the threshold for the selection.

#### 3.3.2. The Critical Road Selection Method

Based on the above analysis, a critical road selection model for traffic state prediction is constructed. In this paper, due to the spatiotemporal state changes of the road network, the selected roads need to be updated at intervals *T*. An improved greedy algorithm is proposed to solve the critical road selection problems. A greedy algorithm means that we always make the best choice for the current situation when solving an optimization problem. In other words, such an algorithm does not consider the overall situation but rather considers only the local situation. The pseudocode of the proposed algorithm is shown in Algorithm 1.

### 3.4. Traffic State Prediction Using the Deep Learning Approach

In this paper, a spatiotemporal recurrent convolutional network is proposed for the prediction (STRCN). The proposed STRCN inherits the advantages of deep convolutional neural networks (DCNN) and long short-term memory (LSTM) neural networks. The spatial dependencies of network-wide traffic can be captured by CNN, and the temporal dynamics can be learned by LSTM.

#### 3.4.1. Capturing Spatial Features by CNN

CNN has been successfully applied to traffic prediction for its great potential in extracting features using multiple layers. A typical CNN mainly comprises multiple convolution layers and pooling layers. The former contributes to mine spatial dependencies of road sections since every layer retrieves a distinct feature using different filters. In comparison, the latter assists in reducing the number of parameters required for training CNN under the premise of ensuring prediction accuracy. Given that the input for CNN could be intuitively regarded as an image with each pixel value associating one kind of traffic state during a certain time, 2D CNN is naturally utilized to abstract spatial features between road sections.  Figure 2 illustrates the structure of CNN, including the input layer, convolution layer, pooling layer, fully connected layer, and output layer. Each part plays a unique and vital role for CNN, and the details are briefly explained below.

Suppose that we need to predict the future traffic speed of the network *V*^*t*+*a*^={*v*_*i*_^*t*+*a*^}_*i*=1_^*m*^, where *a* is the prediction horizon and *m* is the number of road sections. The input of the CNN is the historical traffic speed of critical road sections {*U*^*t*−*n*^, *U*^*t*−1^, *U*^*t*^}, where *U*^*t*−*n*^={*v*_*i*_^*t*−*n*^}_*i*=1_^*P*_*α*_^ represents the traffic state of critical road sections at time (*t*−*n*), *n* is the look back step, and *P*_*α*_ is the number of critical road sections. Then, the spatial features of input are captured by convolutional and pooling layers. Let *O*_*r*_^*l*^ be the output of *l*th convolutional and pooling layers with *r* filters and the weights and bias of *l*th layers be (*W*_*r*_^*l*^, *b*_*r*_^*l*^). Then, the *O*_*r*_^*l*^ could be calculated by the following equation:

(9) $$\begin{array}{c} O_{r}^{l}=\text{pool}\left(f\left(\sum_{r}W_{r}^{l}*O_{r}^{l-1}+b_{r}^{l}\right)\right), \end{array}$$

where *O*_*r*_^*l*−1^ means the output of the previous layer and *O*_*r*_^1^ is exactly the input layer. *f* is a nonlinear activation function, and pool denotes the pooling procedure.

#### 3.4.2. Capturing Temporal Features by LSTM

Intuitively, traffic states at each moment have a strict sequential relationship in time dimension rather than isolated from each other, which is especially suitable for RNN to capture the temporal evolution of traffic flow. However, it is difficult for traditional RNN to capture temporal dependency if two time intervals are remote. Then, LSTM, one of the specific forms of RNNs, is proposed to tackle these issues by adding memory cells in hidden layers. As shown in Figure 3, four main parts, an input gate, a neuron with a self-recurrent connection, a forget gate, and an output gate, are collaborated to alleviate the problems of traditional RNN caused by the gradient vanish and explosion.

In our model, next to CNN, the LSTM naturally takes the output of CNN *V*^*t*^={*x*_*i*_^*t*^}_*i*=1_^*R*^ as its input to predict the future traffic states *H*_*t*_={*h*_*i*_^*t*^}_*i*=1_^*q*^, namely, its output, where *q* is the number of hidden units of the output layer. For a memory cell, the input states are *G*_*t*−1_ while the output is *G*_*t*_. Meanwhile, the states of input, forget, and output gates are *I*_*t*_, *F*_*t*_, and *O*_*t*_, respectively. The temporal features could be iteratively calculated by the following equations:

(10) $$\begin{array}{c} \text{input gate}:I_{t}=\sigma \left(W_{v}^{i}V^{t}+W_{h}^{i}H^{t-1}+b_{i}\right), \end{array}$$

(11) $$\begin{array}{c} \text{forget gate}:F_{t}=\sigma \left(W_{v}^{f}V^{t}+W_{h}^{f}H^{t-1}+b_{f}\right), \end{array}$$

(12) $$\begin{array}{c} \text{output gate}:O_{t}=\sigma \left(W_{v}^{O}V^{t}+W_{h}^{o}H^{t-1}+b_{o}\right), \end{array}$$

(13) $$\begin{array}{c} \text{cell input}:G_{t-1}=\tanh\left(W_{v}^{c}V^{t}+W_{h}^{c}H^{t-1}+b_{c}\right), \end{array}$$

(14) $$\begin{array}{c} \text{cell output}:G_{t}=I_{t}⊙G_{t}+F_{t}⊙G_{t-1}, \end{array}$$

(15) $$\begin{array}{c} \text{hidden layer output}:H_{t}=O_{t}⊙\;\tanh\left(G_{t}\right), \end{array}$$

where weights matrices *W* and bias vectors *b* are constructed to connect input layer, output layer, and the memory cell, ⊙ denotes the scalar product of two vectors, and *σ*(·) represents the standard logistics sigmoid function defined as follows:

(16) $$\begin{array}{c} \sigma \left(x\right)=\frac{1}{1+e^{-x}}. \end{array}$$

#### 3.4.3. Training with STRCN

Integrated with the advantages of CNN and LSTM, the STRCNs is utilized to predict future traffic states by sufficiently exploiting the spatiotemporal characteristics of the data. Eventually, a fully connected layer is employed to predict the future speed by taking the output of LSTM as input. The future speed could be calculated by the following equation:

(17) $$\begin{array}{c} Y^{t+1}=W_{y}H_{t}+b_{y}, \end{array}$$

where *W*_*y*_ and *b*_*y*_ are weight and bias related to the hidden layer. Conclusively, the model is trained from end to end, and the values of *Y*^*t*+1^ are prediction results, which are the output of the entire mode. Several hyperparameters within the model will be set and elaborated in the experiment section. Additionally, it is significant to note that the input size will alter as the number of critical road sections changes due to different extracting rate *α*, and hence several hyperparameters will change too.

## 4. Case Study

### 4.1. Data Used

In this section, a case study is conducted to evaluate the performance of the proposed critical road selection optimization model and the traffic prediction method. The main urban road of a subtransportation network of Beijing near West Second Ring Road is selected as the research objective, as shown in Figure 4. The network comprises 278 road sections, including several kinds of hierarchies of roads, such as freeways, arterials, secondary roads, and collectors. The total length of all the roads is approximately 24.53 km, and the network covers around 0.6 km^2^ areas.

Data collected by taxis equipped with GPS devices from June 1st, 2015, to August 31st, 2015 (92 days) is utilized for training the proposed model and predicting the future traffic speed of the network. The updating frequency of data is 2 minutes, and a time period ranging from 6 : 00 : 00 to 23 : 00 : 00 is concerned for high travel demand is repeatedly observed. Accounting for the traffic state varies every time interval, we could observe 511 traffic states per day.

### 4.2. Critical Road Selections

The proposed QoS-based critical road selection method and other two road selection methods (random method and coverage-based method) were used to select the road sections for prediction in the road network. In a random method, the road is selected randomly during the prediction process. In the coverage-based method, the road is selected based on the coverage, which means that roads with higher coverage are preferred for selection. The three critical road selection methods are applied under different roads extracting rate *μ* (i.e., the proportion of critical road sections to all roads, *μ* ∈ [10%, 20%,  30%,  40%, 50%, 60%, 70%, 80%, 90%, 100%]).

Eventually, the correspondence of extracting rate and the number of critical road sections are listed in Table 1. For example, *μ*=0.50 means that we will select 139 roads as critical road sections and subsequently use them to predict the traffic states of 278 roads.

### 4.3. Results and Comparison

#### 4.3.1. Performance between Different Critical Road Selection Methods

The root means squared error (RMSE) and root mean squared error proportional (RMSEP) are employed to evaluate the performance of all the models, which could be calculated as in the following equations:

(18) $$\begin{array}{c} \text{RMSE}=\frac{1}{n_{\mu }}\sqrt{n_{\mu }\sum_{i=1}^{N_{\mu }}{\left({\hat{y}}_{i}-y_{i}\right)}^{2}}, \end{array}$$

(19) $$\begin{array}{c} \text{RMSEP}=\frac{100}{{\hat{y}}_{i}^{\text{ave}}}\sqrt{\frac{1}{n_{\mu }}\sum_{i=1}^{N_{\mu }}{\left({\hat{y}}_{i}-y_{i}\right)}^{2}}, \end{array}$$

where ${\hat{y}}_{i}$ is the *i*th ground-truth value and *y*_*i*_ is the *i*th predicted value. The value of *n*_*μ*_ denotes the number of critical road sections at extracting rate *μ* and *N*_*μ*_ is the total number of traffic states.

#### 4.3.2. Performance Using the Different Critical Road Selection Method

In order to evaluate the performance of the proposed critical road selection optimization model, we train and test the STRCN model using different road selection methods. The RMSEs and RMSEPs in the context of different extracting rates *μ* are listed in Table 2.

It could be found that in the range of 0.8 to 1.0, the performance of the STRCN model using different road selection methods is almost the same. The reason is that the finally selected road sections by different methods have little difference under the condition of high extracting rate. However, when the extracting rate is between 0.5 and 0.8, the performance of the QoS-based selection method is a little superior to the overall prediction model. In general, the decrease of accuracy is reasonable and within the acceptable limits, which demonstrates the validation and generalization of the approach and the fact that some road sections indeed have less contribution towards prediction.

Additionally, when the extracting rate comes to 0.5, the predictive performance gradually tends to be unstable, probably because too many roads are omitted. Particularly when the extracting rate is between 0.0 and 0.2, the performance is basically the same. That is because no matter what method is used, there are too many missing road sections to predict.  Figure 5 shows that prediction accuracy generally declines as the extracting rate decreases with different critical road selection methods.

#### 4.3.3. Performance between Several DL Algorithms

As we introduced before, corrupted or missing data generally exist on account of the monitoring equipment failure, extreme weather, data transmission error etc., which weakens the effectiveness of the prediction model or even disables the model. To test the performance of our model under random structural missing data, we stochastically extract a part of road sections of the rate of *μ* where the value remains the same as those mentioned above.

Four popular deep learning-based algorithms are selected for comparison, including ANN, CNN, LSTM, and SAE. ANN adopts a plain and shallow structure to process multidimension and nonlinear problems. The parameters of the SAE are set according to [35], which achieves high accuracy in predicting traffic flow. We take 30 min historical traffic speed as the input to predict overall traffic states after 2 min.

Table 3 presents the quantitative results of Q-STRCN, ANN, CNN, and LSTM. It could be observed that the result of Q-STRCN outperforms other models, indicating that our model could precisely mine the spatiotemporal features of the data and make a relatively accurate prediction. Among all the rival algorithms, LSTM has the best performance, probably resulting from that the temporal features of the time-series data are essentially prominent. The results of ANN and SAE demonstrate that these two models fail to extract spatiotemporal characteristics that have vital impacts on prediction.  Figure 6 shows the quantitative results among different approaches under different extracting rates.

## 5. Summary and Conclusions

Structural missing data usually has a massive negative effect on short-term traffic state prediction. In this paper, a novel hybrid short-term traffic state prediction method based on critical road selection optimization is proposed. First, the utility function of the quality of service (QoS) for the critical roads in a large-scale road network is proposed based on the coverage and the data score. Then, the critical road selection optimization model in the transportation networks is presented by selecting an appropriate set of critical roads with the maximum proportion of the total calculation resources to maximize the utility value of the QoS. Also, an innovative critical road selection method, which is considering the topological structure and the mobility of the urban road network, is introduced. Subsequently, the traffic speed of the critical roads is regarded as the input of the convolutional long short-term memory neural network to predict the future traffic states of the entire network. Experiment results on the Beijing traffic network indicate that the proposed method outperforms prevailing DL approaches in the cases of considering critical road sections.

However, even the case study showed that the proposed method could significantly improve the QoS of the traffic prediction, there is still a long way to go from practical application for the method. For future studies, the inherent attributes of the road should be taken into account when calculating the QoS for the road network. Besides, the traffic accident, temperature, weather, and other external factors affect the traffic prediction accuracy. All these will be left for our future research.

## Figures and Tables

**Figure 1:** An area of the urban road network in Beijing, China. (a) The primal graph of the road network and (b) the gridding of the road network.

**Figure 2:** The structure of the CNN.

**Figure 3:** The architecture of LSTM NN.

**Figure 4:** The layout of the subtransportation network in Beijing.

**Figure 5:** The trend of prediction accuracy using different critical road selection methods. (a) The RMSE of different methods and (b) the RMSEP of different methods.

**Figure 6:** The quantitative results among different approaches under different extracting rates. (a) *μ*=0.8; (b) *μ*=0.7; (c) *μ*=0.6; (d) *μ*=0.5.

**Algorithm 1:** Greedy-based critical road selection method (pseudocode of the proposed algorithm).

**Table 1:** Correspondence of extracting rate and the number of critical road sections.

Parameters	Values								
Extracting rate *μ*	0.60	0.65	0.70	0.75	0.80	0.85	0.90	0.95	1.00
Number of roads	167	181	195	209	222	236	250	264	278

**Table 2:** Performance of the STRCN using different critical road selection methods.

Extracting rate *μ*	QoS-based method		Random method		Coverage-based method	
	RMSE	RMSEP (%)	RMSE	RMSEP (%)	RMSE	RMSEP (%)
1.0	6.767	21.019	6.766	21.013	6.768	21.022
0.9	6.911	21.572	6.901	22.021	6.875	21.531
0.8	7.143	22.698	7.175	22.781	7.144	22.700
0.7	7.144	22.693	7.231	23.276	7.174	23.091
0.6	7.027	21.425	7.285	23.763	7.186	23.113
0.5	7.089	21.889	7.301	24.017	7.197	23.150
0.4	7.179	22.802	7.376	24.172	7.223	23.350
0.3	7.235	23.763	7.405	24.508	7.331	24.003
0.2	7.471	24.078	7.479	24.967	7.474	24.095
0.1	7.701	25.102	7.705	25.109	7.703	25.108

**Table 3:** Performance between several DL algorithms.

*μ*	Q-STRCN		LSTM		CNN		ANN		SAE	
	RMSE	RMSEP	RMSE	RMSEP	RMSE	RMSEP	RMSE	RMSEP	RMSE	RMSEP
0.8	7.143	22.698	7.198	22.701	7.213	23.101	8.173	27.134	7.989	26.311
0.7	7.144	22.693	7.351	22.816	7.939	26.631	9.512	31.781	8.296	28.501
0.6	7.027	21.425	8.136	26.589	8.813	26.897	10.891	36.123	9.375	30.134
0.5	7.089	21.889	9.257	30.317	9.785	30.871	11.231	39.177	10.012	33.891

## Data Availability

All data, models, and code generated or used during the study are available in the submitted article.
